The article "Long non‐coding RNA XIST binding to let‐7c‐5p contributes to rheumatoid arthritis through its effects on proliferation and differentiation of osteoblasts via regulation of STAT3" was retracted in 2021. Reasons: results that could not be reproduced; signs of a paper mill; unreliable results or conclusions.

# Long non‐coding RNA XIST binding to let‐7c‐5p contributes to rheumatoid arthritis through its effects on proliferation and differentiation of osteoblasts via regulation of STAT3

**DOI:** 10.1002/jcla.23496

**Published:** 2020-09-03

**Authors:** Zong‐Qiang Wang, Dian‐Hui Xiu, Jin‐Lan Jiang, Gui‐Feng Liu

**Affiliations:** ^1^ Medical Department China‐Japan Union Hospital of Jilin University Changchun China; ^2^ Department of Radiology China‐Japan Union Hospital of Jilin University Changchun China; ^3^ Department of Orthopedics China‐Japan Union Hospital of Jilin University Changchun China; ^4^ Scientific Research Center China‐Japan Union Hospital of Jilin University Changchun China

**Keywords:** Let‐7c‐5p, long non‐coding RNA X‐inactive specific transcript, osteoblast, rheumatoid arthritis, signal transducer and activator of transcription 3

## Abstract

**Background:**

Rheumatoid arthritis (RA), a chronic autoimmune disease, affects around 1% population worldwide, with the life quality of patients severely reduced. In this study, it is intended to explore the role of long non‐coding RNA X‐inactive specific transcript (lncRNA XIST) in RA and the underlying mechanisms associated with let‐7c‐5p and signal transducer and activator of transcription 3 (STAT3).

**Methods:**

LncRNA XIST, let‐7c‐5p, and STAT3 expressions were determined in RA and normal cartilage tissues, and their relationship was analyzed in osteoblasts. The regulatory effects of lncRNA XIST in RA were investigated when XIST expression was upregulated or downregulated in osteoblasts. TNF‐α, IL‐2, IL‐6, alkaline phosphatase (ALP), osteocalcin, TGF‐β1, and IGF1 were measured in vivo in RA rats.

**Results:**

LncRNA XIST and STAT3 were expressed at high levels and let‐7c‐5p expressed at a low level in RA cartilage tissues. LncRNA XIST silencing or let‐7c‐5p enhancement led to decreased levels of TNF‐α, IL‐2, and IL‐6, suggestive of suppressed inflammatory response, and increased levels of ALP, osteocalcin, TGF‐β1, and IGF‐1 as well as reduced damage in cartilage tissues.

**Conclusion:**

LncRNA XIST downregulation could promote proliferation and differentiation of osteoblasts in RA, serving as a future therapeutic target for RA.

## Graphical abstract

LncRNA XIST downregulation could promote proliferation and differentiation of osteoblasts in RA via the inhibition of STAT3 by increasing the expression of let‐7c‐5p.

## 1 INTRODUCTION

Rheumatoid arthritis (RA) is a chronic and inflammatory disorder, which can result in joint destruction, deformity, and even disability.^1^ However, the etiology and pathogenesis of RA remain unclear, although it has been hypothesized that RA may result from the combined effects of genetic and environmental factors.^2^, ^3^ RA is associated with multiple characteristics, including cartilage degradation, bone erosion, and joint instability.^4^ Nowadays, RA is reported to affect approximately 1% of the world population, while the life quality of RA patients and their life expectancy have both been reduced by this disease.^5^, ^6^ The impact of inflammation in osteoblasts has been proved, which displays crucial roles within the arthritic bone microenvironment, and, thus, in RA pathogenesis.^7^ Although there are some therapies available for the inhibition of inflammation, they only achieved limited efficacy in specific patients.^8^ Thus, it is necessary to find a new therapeutic target for the diagnosis and treatment of RA.

Long non‐coding RNAs (lncRNAs) are defined as a group of RNA transcripts with more than 200 nucleotides in length.^9^ A number of investigations have shown that lncRNAs exert great effects on several inflammatory diseases, including RA.^10^, ^11^ For instance, lncRNA NR024118 serves as a diagnostic biomarker for RA.^12^ Recently, X‐inactive specific transcript (XIST), a newly discovered lncRNA, is identified to be related to the progression of multiple tumors, such as breast cancer and bladder cancer.^13^, ^14^ However, the role of XIST in RA remains unclear. Moreover, the regulatory relationship between lncRNAs and microRNAs (miRs) has been widely recognized.^15^ MiRs are small non‐coding RNA molecules, which function as regulators to inhibit the translation of messenger RNAs (mRNAs) by binding to the 3′ untranslated region (3′UTR) of their target mRNAs.^16^, ^17^ It is also known that miRs play crucial roles in the development of RA.^18^ In particular, as one of the most abundant and highly conserved miRs, let‐7c acts as a suppressor in human cancers by affecting the proliferation and apoptosis of cancer cells.^19^ Additionally, the phosphorylation of signal transducer and activator of transcription 3 (STAT3) has also been implicated in the occurrence of RA.^20^ Let‐7c induced by antrocin treatment has been demonstrated to inhibit STAT3 expression^21^ that has been proved to be associated with osteoblast differentiation.^22^ This study was performed to validate the effect of siRNA‐mediated silencing of lncRNA XIST on the proliferation and differentiation of osteoblasts in a rat model of RA, and the involvement of let‐7c‐5p and STAT3.

## 2 MATERIALS AND METHODS

### 2.1 Ethics statement

All animal experiments were performed in line with the Guide for the Care and Use of Laboratory Animal. Moreover, this study was approved by the Ethics Committee of Clinical Medical College, Yangzhou University, while all patients had provided the signed forms of informed consent.

### 2.2 Establishment of RA rat models

A total of 80 male Wistar rats (weighing 160‐180 g) were purchased from the Animal Experiment Center of Southern Medical University (Guangzhou, Guangdong, China). All rats were housed in a level‐2 clean animal room under 50%‐60% humidity at 22‐24°C. The alternating light and dark periods were set for 12 hours each, and the rats were granted with free access to food and water during 1 week of adaptation. An acetic acid solution of bovine cartilage type II collagen (4 mg/mL) was added into cold Freund's complete adjuvant at a 1:1 ratio for efficient emulsification. Subsequently, each rat was intracutaneously injected with the emulsion (0.25 mL in total) into the left paw, the root of the stomach, and the back. After 7 days, a booster injection of emulsion was given to the right paw, the root of the tail, and the back using the same method above. After the booster injection, the rats showed severely swollen paws, an increase of ≥2 mm in the ankle diameter, and an increase of ≥0.80 mL in the size of rear paw, indicating that the model was successfully established.^23^

Lentiviral vectors were constructed. Target gene sequences were amplified by PCR, and the amplified products were cloned into the overexpression lentiviral vector pLV‐EGFP‐N at the ECOR1 and NOT1 sites using the Cold Fusion kit (SBI Inc.). Cells were transfected with empty lentivirus particles or overexpressed lentivirus particles and selected with puromycin for 3 days to obtain a stable cell line. Both negative control (NC) and short hairpin RNA (shRNA) targeting lncRNA XIST (sh‐lncRNA XIST) were purchased from Gene Pharma (Shanghai, China). Lentiviral packaging was performed in human embryonic kidney (HEK)‐293T (293T) cells. 293T cells were cultured in Roswell Park Memorial Institute 1640 (RPMI‐1640) containing 10% fetal bovine serum (FBS) and passaged every other day. Virus were collected and divided into the NC group and the sh‐lncRNA XIST group according to different transfections.

After successful modeling, rats were anesthetized with 3% pentobarbital sodium (Cat. No.: P3761; Sigma‐Aldrich Chemical Company). Rats were fixed by a sterilizing test bench. The tails of the rats were grasped and scrubbed with alcohol cotton balls. After the veins on both sides of the tail were dilated, the lentiviral vector (1 × 10^7^ IU), let‐7c‐5p agomir, or let‐7c‐5p antagomir (20 nmol/L) was 30° obliquely injected into the dilated tail vein. After 48 hours of infection, GFP expression efficiency was observed by fluorescence microscopy. A total of 80 mice were used in the model establishment. There were 9 dead mice, and 5 mice were excluded due to unsuccessful model establishment. Subsequently, 8 mice from the rest of 66 mice served as the blank group (without any treatment), and 56 mice from the remaining 58 mice were divided into 7 groups (n = 8 in each group): NC (RA rats injected with lentivirus carrying NC plasmids), sh‐lncRNA XIST (RA rats injected with lentivirus carrying sh‐lncRNA XIST plasmids), let‐7c‐5p agomir (RA rats injected with lentivirus carrying let‐7c‐5p agomir), let‐7c‐5p antagomir (RA rats injected with lentivirus carrying let‐7c‐5p antagomir), sh‐lncRNA XIST + let‐7c‐5p antagomir (RA rats injected with lentivirus carrying sh‐lncRNA XIST + let‐7c‐5p antagomir), oe‐STAT3 (RA rats injected with lentivirus carrying STAT3‐overexpressing sequence), and sh‐lncRNA XIST + oe‐STAT3 (RA rats injected with lentivirus carrying sh‐lncRNA XIST and oe‐STAT3) groups. After successful injection of plasmids or lentiviruses, rats were anesthetized with pentobarbital sodium (100 mg/kg) and euthanized.

### 2.3 Study subject

The cartilage tissues in the knee joint were collected from 39 RA patients (average age: 52.92 ± 3.04 years, ranging from 41 to 62 years) who received treatment in the Bone and Joint Center of Clinical Medical College, Yangzhou University, from January 2015 to October 2017. The subjects, including 16 males and 23 females, were enrolled into the experimental group. The RA in these patients has progressed 3‐8 years after its first diagnosis. All patients were diagnosed by clinical and arthroscopic evidence in accordance with the classification standard of American College of Rheumatology (ACR) in 1987. Meanwhile, other 7 cases of cartilage tissues in the knee joint were collected from patients (average age: 43.29 ± 3.864 years, ranging from 37 to 49 years) undergoing amputation as the result of accidents. These 7 subjects, including 5 males and 2 females, were enrolled into the control group. The collected tissues were preserved in liquid nitrogen or in a −80°C freezer for future use. Details of patient information are shown in Table 1.

**Table 1:** Baseline characteristics of the RA patients and healthy people in this study

	RA patients	Healthy people
Age bracket (year)	41‐62	37‐49
Average age (year)	52.92 ± 3.04	43.29 ± 3.86
Gender		
Male	16	5
Female	23	2
Disease course (year)	2019.3.8	0

Abbreviation: RA, rheumatoid arthritis.

### 2.4 RT‐qPCR

The total RNA of cell and tissue samples was extracted using a Trizol kit (15596026; Invitrogen Inc.) and reversely transcribed into cDNA using a PrimeScript RT reagent kit (RR047A; Takara Holdings Inc.). The primer sequences (Table 2) for lncRNA XIST, let‐7c‐5p, STAT3, alkaline phosphatase (ALP), osteocalcin (OCN), transforming growth factor β1 (TGF‐β1), insulin‐like growth factor 1 (IGF1), U6, and glyceraldehyde‐phosphate dehydrogenase (GAPDH) were designed and synthesized by Shanghai Sangon Biotech Co., Ltd. (Shanghai, China). The RT products were collected for real‐time fluorescence quantitative PCR, which was conducted following the instructions of a SYBR^®^Premix Ex Taq™ II kit (Takara Biotechnology Ltd.). An ABI PRISM^®^ 7500 System (ABI Company) was used for real‐time PCR. The relative expression of target genes was calculated based on the 2^−ΔΔ^ *^C^* ^t^ method.^24^

**Table 2:** Primer sequences of related genes for RT‐qPCR

Gene	Forward primer (5′‐3′)	Reverse primer (5′‐3′)
LncRNA XIST (human)	CTCTCCATTGGGTTCAC	GCGGCAGGTCTTAAGAGATGAG
LncRNA XIST(rat)	AGCTCCTCGGACAGCTGTAA	CTCCAGATAGCTGGCAACC
let‐7c‐5p (human)	UGAGGUAGUAGGUUGUAUGGUU	CCAUACAACCUACUACCUCAUU
let‐7c‐5p (rat)	CGTGCGGTGAGGTAGTAGGTT	GTGCAGGGTCCGAGGTATTC
STAT3 (human)	CAGCAGCTTGACACACGGTA	AAACACCAAAGTGGCATGTGA
STAT3 (rat)	ACCTGCAGCAA‐TACCATTGAC	AAGGTGAGGGACTCAAACTGC
ALP	GTGAACCGCAACTGGTACTC	GAGCTGCGTAGCGATGTCC
OCN	CACTCCTCGCCCTATTGGC	CCCTCCTGCTTGGACACAAAG
TGF‐β1	GGCCAGATCCTGTCCAAGC	GTGGGTTTCCACCATTAGCAC
IGF‐1	GCTCTTCAGTTCGTGTGTGGA	GCCTCCTTAGATCACAGCTCC
U6 (human)	CTCGCTTCGGCAGCACA	AACGCTTVAGGAATTTGCGT
U6 (rat)	CTCGCTTCGGCAGCACA	AACGCTTCACGAATTTGCGT
Runx1	TGACAGCATCTGCGAGCGAA	ACTTGCGACTTGGTCCTTG
Osx	TGGGAACACCTCGTAACTAC	CACTCATCACAGTACTTGCCTC‐
Col1al	CAATCTGCCTACCGTGCGTC	GCCTTCTCGCTCGTTCCA
Bglap	GGTCATGAGCCGACCAAGTT	GTCTGCAAGTAGACTCCAGG
GAPDH	GGAGCGAGATCCCTCCAAAAT	GGCTGTTGTCATACTTCTCATGG

Abbreviations: ALP, alkaline phosphatase; GAPDH, glyceraldehyde‐phosphate dehydrogenase; IGF1, insulin‐like growth factor 1; LncRNA XIST, long non‐coding RNA X‐inactive specific transcript; OCN, osteocalcin; RT‐qPCR, reverse transcription quantitative polymerase chain reaction; STAT3, signal transducer and activator of transcription 3; TGF‐β1, transforming growth factor β1.

### 2.5 Western blot analysis

The tissue and cell samples were collected and mixed with a radio‐immunoprecipitation assay (RIPA) lysis buffer (P0013B; Beyotime Biotechnology Co., Ltd.), phenylmethylsulfonyl fluoride (PMSF), and phosphatase inhibitors to collect total protein. Subsequently, 30 µg of total protein was resolved by sodium dodecyl sulfate (SDS)‐polyacrylamide gel electrophoresis (PAGE), transferred onto a nitrocellulose membrane using a wet transfer method, and blocked for 1.5 hours with Tris‐buffered saline and Tween 20 (TBST) containing 5% skimmed milk. The primary rabbit anti‐human antibodies to STAT3 (ab68153, 1:2000), ALP (ab229126, 1:500), OCN (ab93876, 1:500), TGF‐β1 (ab92486, 1:1000), IGF‐1 (ab182408, 1:1000), and GAPDH (ab9485, 1:2500) were incubated with the nitrocellulose membrane at 4°C overnight. On the next day, the membrane was rinsed 3 times with TBST (15 minutes per rinse) and subsequently incubated with horseradish peroxidase (HRP)‐labeled goat anti‐rabbit IgG (ab205718, 1:2000‐1:50 000) at room temperature for 2 hours. After another 3 times of TBST rinsing (15 minutes per rinse), the membrane was subsequently immersed in an electroluminescence (ECL) solution and photographed by a SmartView Pro 2000 system (UVCI‐2100; Major Science). The gray value of protein bands was analyzed using the quantity one software.^25^

### 2.6 Fluorescence in situ hybridization

The coverslips containing migrated cells were placed on the bottom of a 24‐well plate (6 × 10^4^ cells/well). After the cell confluence reached 60%‐70%, the cells were fixed in 4% paraformaldehyde at room temperature for 10 minutes and added with pre‐cooled permeable fluid (1 mL/well) and incubated at 4°C for 5 minutes. Following the removal of the permeable fluid, 20 μL of pre‐hybridization solution was added into each well to block the cells at 37°C for 30 minutes, during which the hybridization solution was preheated to 37°C. The pre‐hybridization solution in each well was then discarded, and hybridization solution containing probes was added. The cells were subsequently hybridized under conditions void of light at 37°C overnight, washed with washing solution I to reduce the background signals at 42°C, and then washed with washing solution II and washing solution III under the same conditions. Subsequently, the samples were stained with a 4′,6‐diamidino‐2‐phenylindole (DAPI) staining solution under conditions void of light for 10 minutes. Finally, cells were fixed on glass slides with a mounting agent prior to fluorescence detection.

### 2.7 Dual luciferase reporter gene assay

The target genes of let‐7c‐5p were predicted using target gene prediction software, and dual luciferase reporter gene assay was performed to verify that lncRNA XIST and STAT3 were direct target genes of let‐7c‐5p. Site‐directed mutagenesis was carried out in the let‐7c‐5p binding sites of wild‐type (WT) 3′ untranslated region (UTR) of STAT3 mRNA and lncRNA XIST, so that mutant (MUT) sequences of lncRNA XIST and STAT3 mRNA were synthesized. Subsequently, a pmiR‐RB‐REPORT™ vector (Guangzhou Ribo Biotechnology Co., Ltd.) was treated with restriction enzymes to insert the synthesized gene fragments of WT and MUT lncRNA XIST and STAT3 mRNA, respectively. Meanwhile, the empty plasmids were used as the control group. The WT and MUT luciferase reporter plasmids were then used for subsequent transfections. After 48 hours of transfection, the cells were collected, lysed, and centrifuged for 3‐5 minutes to collect the supernatant. A Firefly Luciferase Assay Kit (RG005; Beyotime Biotechnology) was used for luciferase activity detection.^26^

### 2.8 RNA immunoprecipitation

A RNA immunoprecipitation (RIP) kit (Millipore Corp.) was used to detect the binding between lncRNA XIST and Argonaute 3 (AGO2) protein. The RA cartilage cells were washed with pre‐cooled PBS, and the supernatant was discarded. An equal amount of RIPA lysis buffer (P0013B, Beyotime Biotechnology) was added into each sample and incubated in an ice bath for 5 minutes to lyse the cells. Subsequently, the cells were centrifuged, followed by the collection of the supernatant. A portion of cell extract was isolated as input, and the remaining part was incubated with antibody for co‐precipitation. Each system (50 μL) of co‐precipitation reaction was washed with magnetic beads and resuspended in 100 μL of a RIP Wash Buffer. The antibody (5 μg) was then added and incubated with the samples for binding. After being rinsed, the bead‐antibody complex was resuspended in 900 μL of RIP Wash Buffer and incubated with 100 μL of cell extract at 4°C overnight. The samples were then placed on a magnet base to collect the bead‐antibody complexes. The samples and input were, respectively, detached with protease K to extract RNA for subsequent PCR detection. The antibody used in RIP was rabbit anti‐human AGO2 (ab186733, 1:50; Abcam Inc.), which was incubated with samples at room temperature for 30 minutes. The rabbit anti‐human IgG (ab109489, 1:100; Abcam Inc.) served as NC.

### 2.9 RNA pull‐down assay

Biotin‐labeled WT‐bio‐let‐7c‐5p and MUT‐bio‐let‐7c‐5p (50 nmol/L, Wuhan GeneCreate Biological Engineering Co., Ltd.) were used to transfect RA cartilage cells. After 48 hours of transfection, the cells were incubated in a specific lysate buffer solution (Ambion) for 10 minutes. The lysate was mixed and incubated at 4°C for 3 hours with M‐280 streptomycin magnetic beads (S3762; Sigma‐Aldrich Chemical Company) pre‐coated with RNase‐free bovine serum albumin and yeast tRNA (TRNABAK‐RO; Sigma‐Aldrich Chemical Company). The beads were then washed two times with a pre‐cooled lysate buffer solution, washed 3 times with a low‐salt buffer solution, and washed one more time with a high‐salt buffer solution. The collected RNA was purified using Trizol, and qPCR was carried out to detect the enrichment of lncRNA XIST.^27^

### 2.10 Osteoblast isolation, culture, and identification

The subchondral bone of osteoarthritis was carefully dissected. Initially, the cartilage tissues were separated from the tibial plateau, and the trabecular bone tissues were separated from subchondral bone plate of inside tibial plateau. The bone blocks were washed 3 times with 128 U/mL gentamicin (Wuhan CUSABIO Co., Ltd.) and subsequently cut into small pieces using a pair of ophthalmic surgical scissors. After being washed 3 times by a serum‐free medium (Gibco Company) to remove the bone marrow, the bone samples were incubated at 37°C for 20 minutes in a Dulbecco minimum essential medium (DMEM)/F12 medium (Gibco Company) containing 1 mg/mL type I collagenase (Gibco Company). The supernatant and the detached cells were then discarded. Subsequently, the medium containing type I collagenase was added for another round of cell detachment that lasted for 20 minutes. The samples were then washed 3 times with a serum‐free medium. The detached bone slices were incubated at 37°C with a DMEM/F12 medium containing 20% FBS in an incubator with 5% CO_2_ and saturated humidity. The medium was changed 1 time every 2 days. When cells migrated from bone slices to culture dish, the samples were further cultured in a medium containing 10% FBS for 4‐6 weeks. When at confluence, the cells were detached with 0.25% trypsin‐0.02% ethylenediaminetetraacetic acid (EDTA). The samples were filtered using a 20‐μm cell mesh to remove bone slices, and a DMEM medium containing 10^−8^ mol/L 1, 25‐hydroxyl vitamin D3 (Sigma‐Aldrich Chemical Company), 50 μg/mL vitamin C, 20 μg/mL proline, and 10% FBS was utilized for cell passage. Finally, the cell morphology was observed under an inverted microscope (DMi8, Leica Biosystems). RT‐qPCR was adopted to detect the expression of osteogenic genes such as Runx1, Osx, Col1al, and Bglap in osteoblasts after 3 weeks of culture. The Alizarin Red S staining was used to detect mineralized nodules after 3 weeks of cell culture.

### 2.11 Cell grouping and transfection

The subchondral bone osteoblasts in the exponential growth phase were inoculated into 6‐well plates at a concentration of 3 × 10^5^ cells/mL. The osteoblasts were divided into the blank (cells without any treatment), NC (cells transfected with NC plasmids), oe‐lncRNA XIST (cells transfected with oe‐lncRNA XIST plasmids), sh‐lncRNA XIST (cells transfected with sh‐lncRNA XIST plasmids), let‐7c‐5p mimic (cells transfected with let‐7c‐5p mimic plasmids), let‐7c‐5p inhibitor (cells treated with let‐7c‐5p inhibitor plasmids), oe‐STAT3 (cells transfected with oe‐STAT3 plasmids), sh‐lncRNA XIST + let‐7c‐5p inhibitor (cells transfected with sh‐lncRNA XIST + let‐7c‐5p inhibitor plasmids), and sh‐lncRNA XIST + oe‐STAT3 (cells transfected with oe‐lncRNA XIST + oe‐STAT3 plasmids) groups. The target plasmids were purchased from Dharmacon. The cells were seeded into 6‐well plates at a density of 3 × 10^5^ cells/mL. When the cell confluence reached 80%, a lipofectamine 2000 (Invitrogen Inc.) kit was used for transfection.

### 2.12 Enzyme‐linked immunosorbent assay

The levels of tumor necrosis factor (TNF)‐α, interleukin (IL)‐2, and IL‐6 were measured using related Enzyme‐linked immunosorbent assay (ELISA) kits (RapidBio Systems, Inc.), respectively. The antigen was diluted using coated diluent at a ratio of 1:20. Each well was added with 100 μL of standard diluent and incubated at 4°C overnight. After the removal of the fluid from the wells, the samples were washed 3 times with washing solution (1 minute per wash), dried using a piece of absorbent paper, and stored at 4°C for future use. The diluted samples were added into reaction wells of an enzyme labeled plate (100 μL/well). The negative and positive controls were set, and detection was conducted in duplicate wells. Subsequently, the fluid in the wells was discarded. The plate was washed 3 times with a washing solution (1 minute per wash) and fully dried using a piece of absorbent paper. Each well was then incubated with 100 μL of diluted enzyme conjugates of the sample at 37°C for 30 minutes. After the plate was washed and dried, the samples were incubated with 100 μL of HRP substrate solution and developed under conditions void of light at 37°C for 10‐20 minutes. When an obvious color change occurred in the positive control, or when a slight color change occurred in the negative control, the reaction in the wells was terminated by 50 μL of terminating liquid. Within 20 minutes, the optical density (OD) value of each well was measured at a wavelength of 450 nm using a microplate reader (SpectraMax M5; Molecular Devices).^28^

### 2.13 Immunofluorescence staining

Cells were collected, seeded on a cover glass, and rinsed three times with PBS (3 minutes per rinse). Subsequently, the cells were fixed with 4% polyoxymethylene, and rinsed three times with PBS (3 minutes per rinse). After being cleared by 0.2% Triton X‐100 at room temperature for 20 minutes, the samples were washed three times with PBS (3 minutes per rinse). Subsequently, the PBS on the glass was dried by absorbent paper, and normal goat serum was added onto the glass to block the samples at room temperature for 30 minutes. After the removal of sealing fluid by absorbent paper, the samples were incubated with Collagen I primary antibody (ab34710, 1:500) at 4°C overnight. After being rinsed four times with phosphate‐buffered saline/Tween (PBST, 3 minutes per rinse), the samples were incubated with goat anti‐rabbit secondary antibody to IgG (ab6717, 1:1000) at 37°C for 1 hour, and rinsed three times with PBST (3 minutes per rinse). The samples were then incubated with DAPI under conditions void of light for 5 minutes and treated with a nucleus counterstaining agent. After being washed four times with PBST (5 minutes per wash), the excessive DAPI was discarded. The samples were then mounted, observed, and photographed under a fluorescence microscope.^29^

### 2.14 Alkaline phosphatase staining

The disinfected coverslips were placed into a 6‐well culture plate, and the cells were inoculated into the plate at a density of 2 × 10^4^ cells/mL. The coverslips containing migrated cells were fixed in 10% neutral formalin at room temperature for 15 minutes. After formalin removal, the samples were incubated with an ALP one‐step staining agent (Pierce) at 37°C for 45 minutes. Subsequently, the staining agent was discarded, and the cells were air‐dried at room temperature overnight. After the culture medium was discarded, 100 μL of Triton X‐100 (2 g/L) was added onto the samples for 3 cycles of freeze‐thawing process. Subsequently, 50 μL of ALP substrate agent containing 1 mmol/L p‐nitrophenyl phosphate (PNPP) and 0.1 mol/L MgCl_2_ was added and reacted with the samples at 37°C for 1 hour, and the reaction was terminated using NaOH (1.25 mol/L). The absorbance (A) value at the wavelength of 405 nm was determined using a microplate reader. The ALP activity was expressed as the Sigma unit: 1 Sigma unit was equal to the enzyme activity of 1 moL p‐nitrophenol in 1 hour.^30^

### 2.15 Observation of physiological changes in rats

The thickness of hind paw was measured. Starting on the 21st day, the thickness of hind paw on the same side was measured using a vernier caliper once a week until the 10th week. Each measurement was repeated 3 times to obtain the mean value. All measurements were independently conducted by two investigators. Starting on the 21st day, the degree of joint swelling in the rats of each group was evaluated twice a week. Each measurement was repeated 3 times to obtain the mean value. The degree of lesion was assessed using a 5‐grade scoring method and the highest score of each limb was 4 points, so that the full score in each rat was 16 points. The specific scoring standards were as follows: 0 point referred to no swelling; 1 point referred to the slight swelling on the toe joint; 2 points referred to the swelling on the toe joint and voix pedis joint; 3 points referred to the swelling on paws below the ankle joint; 4 points referred to the swellings on all limbs including the ankle joints, and a complete loss of functions. After the rats were euthanized via anesthesia, the tissues were cut off at the connection between the upper edge of lateral malleolus and the lower end of the embryo bone, and fixed in formalin for histopathological examination.

### 2.16 Safranin O staining

The obtained cartilage tissues of the ankle joint were fixed in 4% paraformaldehyde for 24 hours, and decalcified by 19% EDTA. Subsequently, the specimens were dehydrated in gradient ethanol, degreased by methanol, and embedded in paraffin using standard procedures. The condylar part was sliced into 8‐μm sections, which were subsequently dewaxed by xylene and hydrated in ethanol. The nuclei were counterstained with hematoxylin for 1‐3 minutes. Subsequently, the samples were washed with running water for 1 minute, differentiated by 1% hydrochloric acid‐ethanol for 30 seconds, washed again with running water for 1 minutes, stained with 0.02% fast green solution for 3 minutes, and immersed in 1% glacial acetic acid to remove the remaining fast green. At last, 1% Safranin O solution was used to stain the samples for 3 minutes. The slices were rinsed with 95% ethanol, dehydrated by anhydrous ethanol, and cleared by xylene. Finally, the cartilage tissues were mounted with neutral gum and the changes in cartilage tissues were observed under the microscope.

### 2.17 Hematoxylin‐eosin staining

Eight‐μm‐thick paraffin sections of cartilage tissues were dewaxed with xylene I for 10 minutes, and xylene II for 5 minutes, following washed with anhydrous alcohol for 1 minute, 95% alcohol for 1 minute, and 85% alcohol for 1 minute. Sections were stained with hematoxylin (Beyotime Biotechnology) for 5 minutes. After being infused with hydrochloric acid‐ethanol and immersed in tap water for 15 minutes, sections were stained with eosin for 2 minutes (Beyotime Biotechnology). Sections were sections were dehydrated with 0.85% alcohol for 20 seconds, 95% alcohol for 1 minute, stained with anhydrous alcohol I for 2 minutes, absolute alcohol II for 2 minutes, and immersed in xylene I for 2 minutes, xylene II for 2 minutes. Sections were sealed with neutral gum, following observed under a microscope light microscopy (DMI3000; Leica).

### 2.18 Statistical analysis

Statistical analysis was performed using the SPSS 22.0 software (IBM Corp., Armonk, NY, USA), and measurement data were expressed as mean ± standard deviation. Unpaired data in compliance with normal distribution and homogeneity between two groups were compared using unpaired *t*‐test, while one‐way analysis of variance (ANOVA) and significant testing were conducted for comparison among multiple groups. Data at different time points were compared by repeated measures ANOVA, followed by Bonferroni post hoc test. Correlation coefficients between lncRNA XIST and let‐7c‐5p expression, and correlation between let‐7c‐5p and STAT3 expression in cartilage tissues of RA were calculated by Pearson's correlation test. A *P* value of <.05 was considered as statistically significant.

## 3 RESULTS

### 3.1 LncRNA XIST and STAT3 are upregulated, while let‐7c‐5p is inhibited in RA cartilage tissues

After 28 days of successful establishment of mice model,^31^ cartilage tissues of normal rats and RA rats were collected. Hematoxylin‐eosin (HE) staining results (Figure 1A) showed that osteoblasts were severely damaged and the number of cells was significantly reduced in cartilage tissues. At the same time, cartilage tissues from healthy individuals and RA patients as well as cartilage tissues from normal rats and RA rats were collected. The expression of lncRNA XIST, STAT3, and let‐7c‐5p in RA and normal cartilage tissues in rats (Figure 1B‐E) and human samples (Figure 1D‐F) was determined using RT‐qPCR and Western blot analysis. Compared with that in normal cartilage tissues, the expression of lncRNA XIST and STAT3 was significantly increased, while the expression of let‐7c‐5p was obviously decreased in RA cartilage tissues (*P* < .05). Correlation analysis between lncRNA XIST and let‐7c‐5p expression, and let‐7c‐5p and STAT3 expression in clinical samples displayed that lncRNA XIST was negatively correlated with let‐7c‐5p expression and let‐7c‐5p was negatively correlated with STAT3 expression. These results indicated that lncRNA XIST and STAT3 might be highly expressed in cartilage tissues of RA, and let‐7c‐5p was poorly expressed in these tissues.

**Figure 1:** LncRNA XIST and STAT3 are upregulated, while let‐7c‐5p is suppressed in RA cartilage tissues. A, the morphological changes in normal and RA cartilage tissues of rats assessed by HE staining (×100); B, the lncRNA XIST and let‐7c‐5p expression and the mRNA level of STAT3 in normal and RA cartilage tissues of rats determined by RT‐qPCR; C, the protein level of STAT3 in normal and RA cartilage tissues of rats determined by Western blot analysis; D, the lncRNA XIST and let‐7c‐5p expression and the mRNA level of STAT3 in normal and RA cartilage tissues of human determined by RT‐qPCR; E, the protein level of STAT3 in normal and RA cartilage tissues of human determined by Western blot analysis; F, correlation analysis between lncRNA XIST and let‐7c‐5p expression in clinical samples of RA; G, correlation analysis between let‐7c‐5p and STAT3 expression in clinical samples of RA. All data were measurement data, expressed as mean ± standard deviation. Unpaired data in compliance with normal distribution and homogeneity between two groups were compared using unpaired *t* test. Correlation coefficients between lncRNA XIST and let‐7c‐5p expression and correlation between let‐7c‐5p and STAT3 expression in cartilage tissues of RA were calculated by Pearson's correlation test. *, *P* < .05 vs the normal group (cartilage tissues of normal rats or RA rates, n = 8; cartilage tissues of healthy people or RA patients, n = 53). LncRNA XIST, long non‐coding RNA X‐inactive specific transcript; STAT3, signal transducer and activator of transcription 3; RA, rheumatoid arthritis; RT‐qPCR, reverse transcription quantitative polymerase chain reaction

### 3.2 LncRNA XIST and STAT3 are highly expressed, but let‐7c‐5p is poorly expressed in osteoblasts

After osteoblasts from primary rats were extracted, type Ⅱ collagenase enzyme digestion and adherent culture methods were used. After 3 weeks of culture, cells were attached to the bottom of the culture flask and the bone fragments were climbed out. Scanning electron microscopy showed that cells were various in shape, which were fusiform, triangular, cubic, or polygonal (Figure 2A).

**Figure 2:** High expression of lncRNA XIST and STAT3 but low expression of let‐7c‐5p was observed in RA cartilage tissues, and lncRNA XIST is mainly expressed in the cytoplasm of osteoblasts. A, primary osteoblast observed under an inverted microscope (×200); B, the expressions of osteogenic genes (Runx1, Osx, Col1al, and Bglap) after 0 h of osteoblast extraction and 3 wk of culture determined by RT‐qPCR assay (*, *P* < .05 vs the 0 wk of culture); C, mineralized nodules after 3 wk of cell culture assessed by Alizarin Red S staining; D, the expression of lncRNA XIST, STAT3, and let‐7c‐5p detected by RT‐qPCR assay; E, the protein expression of STAT3 measured by Western; F, location of lncRNA XIST expression in osteoblasts examined by FISH. All data were measurement data, expressed as mean ± standard deviation. Unpaired data in compliance with normal distribution and homogeneity between two groups were compared using unpaired *t* test. *P < .05 vs 0 wk or the normal group. The experiment was repeated 3 times. FISH, fluorescence in situ hybridization; DAPI, 4′,6‐diamidino‐2‐phenylindole

At the same time, RT‐qPCR assay was applied to determine the expression of osteogenic genes such as Runx1, Osx, Col1al, and Bglap after 0 hour of osteoblast extraction and 3 weeks of culture. The results (Figure 2B) demonstrated that compared with 0 hour of culture after osteoblast extraction, the expression of osteogenic genes including Runx1, Osx, Col1al, and Bglap in osteoblasts was significantly elevated after 3 weeks of culture (all *P* < .05). Besides, large pieces of massive nodules were observed in osteoblasts after 3 weeks of culture, which was typical of calcium (Figure 2C). The above results indicated that the osteoblasts cultured in present experiment sufficiently possessed the expression of osteoblast standard.

The osteoblasts were isolated and identified. The expression of lncRNA XIST, let‐7c‐5p, and STAT3 in osteoblasts was detected by RT‐qPCR assay, and the protein expression of STAT3 in osteoblasts was measured by Western blot analysis. The results (Figure 2D,E) displayed that compared with normal rat osteoblasts., expressions of lncRNA XIST and STAT3 in osteoblasts of RA rats were increased, while the expression of let‐7c‐5p was reduced (*P* < .05).

Fluorescence in situ hybridization (FISH) was used to detect the location of lncRNA XIST expression in osteoblasts. The results (Figure 2F) showed that lncRNA XIST was primarily expressed in the cytoplasm and was poorly expressed in the nucleus of osteoblasts. In the Figures, the red part referred to the lncRNA XIST and the blue part represented the nucleus. These findings indicated that lncRNA XIST was primarily expressed in the cytoplasm of osteoblasts.

### 3.3 LncRNA XIST binds to let‐7c‐5p to regulate STAT3 expression

The online prediction software (https://cm.jefferson.edu/rna22/Interactive/) predicted the binding between let‐7c‐5p and lncRNA XIST (Figure 3A) as well as between let‐7c‐5p and STAT3 3′UTR (Figure 3B), suggesting that lncRNA XIST and STAT3 were target genes of let‐7c‐5p. The regulatory relationship between XIST/STAT3 and let‐7c‐5p was further verified by dual luciferase reporter gene assay. Compared with that in the NC group, the luciferase activity of lncRNA XIST‐WT plasmids was significantly inhibited in the let‐7c‐5p mimic group (*P* < .05), but no difference was found in the luciferase activity of lncRNA XIST‐MUT plasmids (*P* > .05). Compared with that in the NC group, the luciferase activity of STAT3‐WT in the let‐7c‐5p mimic group was significantly inhibited (*P* < .05), but no difference was found for STAT3‐MUT plasmids (*P* > .05), suggesting a targeting relationship between let‐7c‐5p and STAT3 (Figure 3C,D).

**Figure 3:** LncRNA XIST binds to let‐7c‐5p to regulate STAT3 expression. A, the binding site between let‐7c‐5p and lncRNA XIST; B, the binding site between let‐7c‐5p and STAT3; C, luciferase activity to verify the relationship between let‐7c‐5p and lncRNA XIST (*, *P* < .05 vs the NC group); D, luciferase activity to verify the relationship between let‐7c‐5p and STAT3 (*, *P* < .05 vs the NC group); E, RIP showed that lncRNA XIST could bind to AGO2 (*, *P* < .05 vs the IgG); F, RNA pull‐down assay showed that lncRNA XIST could directly bind to let‐7c‐5p (*, *P* < .05 vs the NC group); G, the expression of lncRNA XIST, let‐7c‐5p, and STAT3 determined by RT‐qPCR assay after overexpression of lncRNA XIST or let‐7c‐5p in osteoblasts; H, the protein expression of STAT3 measured by Western blot analysis after overexpression of lncRNA XIST or let‐7c‐5p in osteoblasts (*, *P* < .05 *vs*. the NC group). All data were expressed as mean ± standard deviation. Unpaired data in compliance with normal distribution and homogeneity between two groups were compared using unpaired *t* test. Comparisons among multiple groups were conducted by one‐way ANOVA with Tukey's post hoc test. NC, negative control; RIP, RNA immunoprecipitation; WT, wild type; MUT, mutant

Moreover, the RIP and RNA pull‐down assays were used to further verify the correlation between lncRNA XIST and let‐7c‐5p. The results of RIP (Figure 3E) revealed that the anti‐AGO2 antibody could precipitate lncRNA XIST, indicating that lncRNA XIST could form a complex with AGO2, which could then specifically bind to let‐7c‐5p. Additionally, the results of RNA pull down assay (Figure 3F) displayed that as compared with the MUT‐let‐7c‐5p and Bio‐NC groups, the relative enrichment of lncRNA XIST was increased in the WT‐let‐7c‐5p group (*P* < .05). Therefore, lncRNA XIST could specifically bind to let‐7c‐5p and regulate its expression. After overexpressing of lncRNA XIST or let‐7c‐5p in RA rat osteoblasts, RT‐qPCR was adopted to examine lncRNA XIST, let‐7c‐5p, and STAT3 mRNA expression, and Western blot analysis was used to determine STAT3 protein expression (Figure 3G, H). The results suggested that in comparison with the oe‐NC group, lncRNA XIST, STAT3 mRNA, and protein expression were significantly elevated in the oe‐lncRNA XIST group, accompanied by decreased let‐7c‐5p expression (*P* < .05), while the expression of let‐7c‐5p was significantly increased in the let‐7c‐5p mimic group but the STAT3 mRNA and protein expression were significantly decreased ((*P* < .05). The above results confirmed that lncRNA XIST could competitively bind to let‐7c‐5p, thereby positively regulating STAT3 expression.

### 3.4 Silencing of lncRNA XIST or the upregulation of let‐7c‐5p inhibits inflammatory responses in osteoblasts

The extracted primary osteoblasts were identified. After 48 hours of transfection, ELISA was performed to measure the levels of TNF‐α, IL‐2, and IL‐6 in primary osteoblasts, and to investigate the effects of lncRNA XIST and let‐7c‐5p on the inflammatory responses in RA. As shown in Figure 4, there was no obvious difference between the blank and NC groups regarding the levels of TNF‐α, IL‐2, and IL‐6 (all *P* > .05). Compared with the blank and NC groups, the let‐7c‐5p mimic and sh‐lncRNA XIST groups showed significantly lower levels of TNF‐α, IL‐2, and IL‐6, while the let‐7c‐5p inhibitor and the oe‐STAT3 groups displayed an opposite trend (all *P* < .05). Furthermore, the sh‐lncRNA XIST + let‐7c‐5p inhibitor and the sh‐lncRNA XIST + oe‐STAT groups showed no evident difference regarding the levels of TNF‐α, IL‐2, and IL‐6 versus the blank and NC groups (all *P* > .05). In comparison with the sh‐lncRNA XIST group, levels of TNF‐α, IL‐2, and IL‐6 were notably elevated in the sh‐lncRNA XIST + let‐7c‐5p inhibitor and the sh‐lncRNA XIST + oe‐STAT groups (*P* < .05). These findings indicated that the silencing of lncRNA XIST and the upregulation of let‐7c‐5p both inhibited inflammatory responses in osteoblasts, which was reversed by silencing of let‐7c‐5p or overexpression of STAT3.

**Figure 4:** Downregulation of lncRNA XIST and the overexpression of let‐7c‐5p both inhibit inflammatory responses in osteoblasts of RA. All data were measurement data, expressed as mean ± standard deviation. Comparisons among multiple groups were conducted by one‐way ANOVA with Tukey's post hoc test.; *, *P* < .05 vs the blank or NC group; ^#^, *P* < .05 vs the sh‐lncRNA XIST group. ELISA, Enzyme‐linked immunosorbent assay; IL, interleukin; TNF‐α, tumor necrosis factor α

### 3.5 Silencing of lncRNA XIST and upregulation of let‐7c‐5p both promote expressions of osteogenic‐related genes

To investigate the role of lncRNA XIST and let‐7c‐5p in the osteogenesis during RA, RT‐qPCR (Figure 5C) and Western blot analysis (Figure 5A,B) were performed to determine the expression and protein expression of genes related to osteogenesis. There was no obvious difference regarding the expression and protein expression of let‐7c‐5p, lncRNA XIST, STAT3, ALP, OCN, TGF‐β1, and IGF‐1 between the blank and NC groups (all *P* > .05). Compared with the blank and NC groups, the let‐7c‐5p mimic and sh‐lncRNA XIST groups showed significantly elevated levels of let‐7c‐5p and osteogenesis‐related genes (ALP, OCN, TGF‐β1, and IGF‐1) yet decreased levels of lncRNA XIST and STAT3, while the let‐7c‐5p inhibitor group displayed reduced level of let‐7c‐5p, the let‐7c‐5p inhibitor and the oe‐STAT3 groups showed a decrease in levels of osteogenesis‐related genes (ALP, OCN, TGF‐β1, and IGF‐1), accompanied by an increase of STAT3 expression (all *P* < .05). In addition, the sh‐lncRNA XIST + let‐7c‐5p inhibitor and sh‐lncRNA XIST + oe‐STAT3 groups showed no evident difference when compared with the blank and NC groups (all *P* > .05). There were lower expressions of osteogenesis‐related genes (ALP, OCN, TGF‐β1, and IGF‐1) in the sh‐lncRNA XIST + let‐7c‐5p inhibitor and sh‐lncRNA XIST + oe‐STAT3 groups in comparison with the sh‐lncRNA XIST group (*P* < .05). These data suggested that the silencing of lncRNA XIST and the upregulation of let‐7c‐5p both promoted the osteogenesis‐related gene expressions, which was abolished by silencing of let‐7c‐5p or overexpression of STAT3.

**Figure 5:** Silencing of lncRNA XIST and the upregulation of let‐7c‐5p both promote osteogenesis. A, the gray value of STAT3 ALP, OCN, TGF‐β1, and IGF‐1 protein bands in response to the treatment of sh‐lncRNA XIST, let‐7c‐5p mimic, let‐7c‐5p inhibitor, and sh‐lncRNA XIST + let‐7c‐5p inhibitor determined by Western blot analysis; B, the protein levels of STAT3, ALP, OCN, TGF‐β1, and IGF‐1 in response to the treatment of sh‐lncRNA XIST, let‐7c‐5p mimic, let‐7c‐5p inhibitor, and sh‐lncRNA XIST + let‐7c‐5p inhibitor determined by Western blot analysis; C, the lncRNA XIST and let‐7c‐5p expression and the mRNA levels of STAT3, ALP, OCN, TGF‐β1, and IGF‐1 in response to the treatment of sh‐lncRNA XIST, let‐7c‐5p mimic, let‐7c‐5p inhibitor, and sh‐lncRNA XIST + let‐7c‐5p inhibitor determined by RT‐qPCR. All data were measurement data, expressed as mean ± standard deviation. Comparisons among multiple groups were conducted by one‐way ANOVA with Tukey's post hoc test; *, *P* < .05 vs the blank or NC group; ^#^, *P* < .05 vs the sh‐lncRNA XIST group. ALP, alkaline phosphatase; OCN, osteocalcin; TGF‐β1, transforming growth factor β1; IGF1, insulin‐like growth factor 1; GAPDH, glyceraldehyde‐phosphate dehydrogenase

### 3.6 Silencing of lncRNA XIST and the upregulation of let‐7c‐5p both elevate the level of type I collagen protein

Immunofluorescence staining was used to measure the level of type I collagen protein in subchondral bone osteoblasts collected from RA subjects following the loss‐ and gain‐of‐function experiments of lncRNA XIST and let‐7c‐5p. There were red fluorescence signals in the cytoplasm, indicating that type I collage protein was positively stained in the cells (Figure 6A). The positive rate of type I collage protein = the number of positive cells with type I collage protein expression/the total number of cells × 100%. The results showed no obvious difference between the blank and NC groups in terms of the positive rate of type I collagen protein (*P* > .05; Figure 6B). The positive rate of type I collagen protein was much higher in the let‐7c‐5p mimic and sh‐lncRNA XIST groups and lower in the let‐7c‐5p inhibitor group than in the blank and NC groups (*P* < .05), while no difference was detected in the sh‐lncRNA XIST + let‐7c‐5p inhibitor and sh‐lncRNA XIST + oe‐STAT3 groups (*P* > .05). Compared with the sh‐lncRNA XIST group, the expression of type I collagen protein was diminished in the sh‐lncRNA XIST + let‐7c‐5p inhibitor and sh‐lncRNA XIST + oe‐STAT3 groups (*P* < .05). These findings indicated that the silencing of lncRNA XIST and the upregulation of let‐7c‐5p both enhanced the expression of type I collagen protein, which could be reversed by silencing of let‐7c‐5p or upregulation of STAT3.

**Figure 6:** The silencing of lncRNA XIST and the upregulation of let‐7c‐5p both increase the positive rate of type I collagen protein. A, immunofluorescence staining of type I collagen as observed under a microscope (×200); B, positive rate of type I collagen protein in response to the treatment of sh‐lncRNA XIST, let‐7c‐5p mimic, let‐7c‐5p inhibitor, and sh‐lncRNA XIST + let‐7c‐5p inhibitor; all data were measurement data, expressed as mean ± standard deviation. Comparisons among multiple groups were conducted by one‐way ANOVA with Tukey's post hoc test; *, *P* < .05 vs the blank group or NC group; ^#^, *P* < .05 vs the sh‐lncRNA XIST group

### 3.7 Silencing of lncRNA XIST and the upregulation of let‐7c‐5p both enhance ALP activity

Alkaline phosphatase staining was performed to detect the ALP activity of subchondral bone osteoblasts collected from RA samples of different groups treated by lncRNA XIST or let‐7c‐5p. The blue ALP particles appeared in the cytoplasm, demonstrating the positive staining of ALP (Figure 7A). The positive rate of ALP staining = the number of ALP‐positive cells/the total number of cells × 100%. The results (Figure 7B) showed no obvious difference between the blank and NC groups in terms of the ratio of ALP positive cells (*P* > .05). Compared with the blank and NC groups, the number of ALP positive cells was higher in the let‐7c‐5p mimic and sh‐lncRNA XIST groups, and lower in the let‐7c‐5p inhibitor and the oe‐STAT3 groups (*P* < .05). No difference was seen in the sh‐lncRNA XIST + let‐7c‐5p inhibitor and the sh‐lncRNA XIST + oe‐STAT3 groups in comparison with the blank and NC groups (*P* > .05). Compared with the sh‐lncRNA XIST group, the expression of ALP activity in the sh‐lncRNA XIST + let‐7c‐5p inhibitor and sh‐lncRNA XIST + oe‐STAT3 groups was reduced (*P* < .05). The above results suggested that the silencing of lncRNA XIST and the upregulation of let‐7c‐5p both promoted ALP activity, which could be abolished by silencing of let‐7c‐5p or upregulation of STAT3.

**Figure 7:** The silencing of lncRNA XIST and the upregulation of let‐7c‐5p both enhance ALP activity. A, ALP staining results of subchondral bone osteoblasts in RA (× 200); B, the ratio of ALP positive cells in response to the treatment of sh‐lncRNA XIST, let‐7c‐5p mimic, let‐7c‐5p inhibitor, and sh‐lncRNA XIST + let‐7c‐5p inhibitor. All data were measurement data, expressed as mean ± standard deviation. Comparisons among multiple groups were conducted by one‐way ANOVA with Tukey's post hoc test; *, *P* < .05 vs the blank group or NC group; ^#^, *P* < .05 vs the sh‐lncRNA XIST group

### 3.8 Silencing of lncRNA XIST and the upregulation of let‐7c‐5p both ameliorate the pathological state of RA rats

After 21 days of transfection, the mRNA expressions of lncRNA XIST, let‐7c‐5p, and STAT3 in tissues of the foot of mice were examined by RT‐qPCR assay. The protein expression of STAT3 in tissues of the foot was determined by Western blot analysis. The results (Figure 8A,B) demonstrated that the expression of lncRNA XIST was significantly reduced in the sh‐lncRNA XIST group, the expression of let‐7c‐5p was significantly increased, and the mRNA and protein expression of STAT3 was significantly decreased in the sh‐lncRNA XIST and the let‐7c‐5p agomir groups compared with the blank group and the NC group (all *P* < .05), but let‐7c‐5p antagomir group showed a significant decrease in let‐7c‐5p expression and a significant increase in mRNA and protein expression of STAT3 (both *P* < .05).

**Figure 8:** The silencing of lncRNA XIST and the upregulation of let‐7c‐5p both improve the pathological state of RA rats. A, the mRNA expression of lncRNA XIST, let‐7c‐5p, and STAT3 in tissues of the rat foot determined by RT‐qPCR assay; B, the protein expression of STAT3 in tissues of the rat foot measured by Western blot analysis; C, the degree of swelling in RA rats in response to the treatment of sh‐lncRNA XIST, let‐7c‐5p mimic, let‐7c‐5p inhibitor, and sh‐lncRNA XIST + let‐7c‐5p inhibitor; D, paw thickness in response to the treatment of sh‐lncRNA XIST, let‐7c‐5p mimic, let‐7c‐5p inhibitor, and sh‐lncRNA XIST + let‐7c‐5p inhibitor; E, arthritis scores for the degree of swelling in response to the treatment of sh‐lncRNA XIST, let‐7c‐5p mimic, let‐7c‐5p inhibitor, and sh‐lncRNA XIST + let‐7c‐5p inhibitor. All data were measurement data, expressed as mean ± standard deviation. Comparisons among multiple groups were conducted by one‐way ANOVA with Tukey's post hoc test. Data at different time points were compared by repeated measures ANOVA, followed by Bonferroni post hoc test; *, *P* < .05 vs. the blank or NC group

The thicknesses of hind paw on the right side of rats in each group were measured once a week, and the joints of limbs in the rats were graded based on their inflammation for consecutive 8 weeks. The results depicted in Figure 8C,D, and no significant difference in paw thickness and the degree of swelling was observed between the blank and NC groups (both *P* > .05). Compared with the blank and NC groups, the paw thickness and the degree of swelling in RA rats were ameliorated in the let‐7c‐5p agomir and sh‐lncRNA XIST groups, but were aggravated in the let‐7c‐5p antagomir and oe‐STAT3 groups (both *P* < .05). No significant difference was observed in the sh‐lncRNA XIST + let‐7c‐5p antagomir and sh‐lncRNA XIST + oe‐STAT3 groups compared with the blank and NC groups (both *P* > .05). Taken together, the silencing of lncRNA XIST and the upregulation of let‐7c‐5p could both ameliorate the paw thickness and the degree of swelling in RA rats.

### 3.9 Silencing of lncRNA XIST and the upregulation of let‐7c‐5p both improve the degree of cartilage tissue damage in RA rats

Safranin O staining was used to detect the degree of cartilage tissue damage in RA rats following lncRNA XIST and let‐7c‐5p intervention. As illustrated in Figure 9A, the cartilage tissues of rats in the blank and NC groups displayed the most severe cartilage defect, with the presence of a large number of necrotic cartilage cells, a low number of Safranin O stained cells, subchondral tidal line defect, stroma disorder, and randomly distributed cells. Compared with the blank and NC groups, the cartilage of rats in the let‐7c‐5p agomir and sh‐lncRNA XIST groups showed a relatively complete surface structure, with the presence of many more cartilage cells, near normal cartilage structure, and a clear subchondral tidal line. In contrary, the cartilage of rats in the let‐7c‐5p antagomir and oe‐STAT3 groups was severely damaged, with parts of the cartilage completely disappeared and the presence of a large number of necrotic cartilage cells. There were also signs of nuclear eosinophilic staining, severe infiltration of inflammatory cells, disappeared subchondral tidal line, almost no Safranin O staining, and much fewer cartilage cells. Furthermore, no significant difference was observed in the sh‐lncRNA XIST + let‐7c‐5p antagomir and sh‐lncRNA XIST + oe‐STAT3 groups compared with the blank and NC groups (*P* > .05). Based on these results, it was concluded that the silencing of lncRNA XIST and the upregulation of let‐7c‐5p could both ameliorate the degree of cartilage tissue damage in RA rats.

**Figure 9:** The downregulation of lncRNA XIST and the overexpression of let‐7c‐5p both ameliorate the degree of cartilage tissue damage in RA rats. A, images of cartilage tissues of rats after stained with Safranin O staining (×200); B, images of cartilage tissues of rats after stained with HE staining (×100); C, the expression of TNF‐α, IL‐2, and IL‐6 cytokines in serum of rats examined by ELISA. All data were measurement data, expressed as mean ± standard deviation. Comparisons among multiple groups were conducted by one‐way ANOVA with Tukey's post hoc test; *, *P* < .05 vs the blank or NC group

Hematoxylin‐eosin staining results (Figure 9B) showed that the blank, NC, and sh‐lncRNA XIST + let‐7c‐5p antagomir groups displayed infiltration of inflammatory cells, cartilage damage, and severe osteoblast damage, with the presence of a large number of necrotic cartilage cells, but the conditions were relative eased in the let‐7c‐5p agomir and sh‐lncRNA XIST groups. There was the most severe infiltration of inflammatory cells, cartilage damage and osteoblast damage in the let‐7c‐5p antagomir and oe‐STAT3 groups. No significant difference was found in the sh‐lncRNA XIST + let‐7c‐5p antagomir and sh‐lncRNA XIST + oe‐STAT3 groups (*P* > .05).

The levels of TNF‐α, IL‐2, and IL‐6 cytokines in the serum were assessed by ELISA. The results (Figure 9C) suggested that there was no significant difference in the levels of TNF‐α, IL‐2, and IL‐6 between the blank and NC groups (*P* > .05). Compared with the blank group and the NC groups, the levels of TNF‐α, IL‐2, and IL‐6 were significantly decreased in the let‐7c‐5p agomir group and sh‐lncRNA XIST groups (all *P* < .05), which was elevated in the let‐7c‐5p antagomir and oe‐STAT3 groups (all *P* < .05). No significant difference was found in the sh‐lncRNA XIST + let‐7c‐5p antagomir and sh‐lncRNA XIST + oe‐STAT3 groups (*P* > .05). These results collectively demonstrated that silencing lncRNA XIST or overexpressing of let‐7c‐5p downregulated the expressions of cytokine‐related genes.

## 4 DISCUSSION

As a chronic autoimmune disease of the synovium, RA results in severe joint damages.^32^ It has been reported that the clinical course of RA fluctuates and its prognosis is unpredictable.^33^ In recent years, lncRNAs have been identified to play vital roles in RA.^34^ However, the specific mechanism of lncRNA XIST in RA remains poorly understood. Therefore, the present study was designed to test the hypothesis that silencing of lncRNA XIST could promote the proliferation and differentiation of osteoblasts in RA via STAT3 by activating let‐7c‐5p.

At first, the present study demonstrated that lncRNA XIST and STAT3 expressions were upregulated, while let‐7c‐5p expression was downregulated in RA cartilage tissues, and lncRNA XIST negatively regulated let‐7c‐5p expression. Dysregulated expression of lncRNAs is closely related to the progression of many diseases, such as intervertebral disk degeneration, osteoarthritis, and fracture healing.^35^, ^36^ Sun et al^37^ have indicated that the expression of lncRNA XIST is upregulated in non‐small cell lung cancer. In addition, a previous study has revealed the elevation in lncRNA XIST expression in myocardial I/R injury.^38^ Moreover, lncRNA XIST is reported to be negatively correlated with miR‐449a expression.^39^ Accumulating evidence has suggested that the deregulation of miRs exerts great effects on the development and progression of RA.^40^ For example, let‐7c‐5p expression is decreased in breast cancer tissues.^41^ Interestingly, the upregulation of STATs caused by pro‐inflammatory cytokines or growth factors is conductive to the pathogenesis of RA.^42^ Besides, multiple lines of evidences have revealed that high expression of STAT3 contributes to the development of RA.^43^, ^44^, ^45^ More importantly, previously conducted study has suggested lncRNA XIST upregulates STAT3 to facilitate the development of retinoblastoma through binding with miR‐124.^46^ All these findings provided strong support for our results that lncRNA XIST bound to let‐7c‐5p to upregulate STAT3 expression in RA.

Secondly, the findings of our study implied that the silencing of lncRNA XIST and the upregulation of let‐7c‐5p both downregulated the levels of TNF‐α, IL‐2, and IL‐6, thus reducing the level of inflammatory responses. It is well acknowledged that RA is an inflammatory disease.^47^ Pro‐inflammatory cytokines, including TNF‐α and IL‐6, exert great effects on the development of chronic inflammation and joint destruction.^48^, ^49^ In recent years, emerging evidence has supported the crucial role of lncRNA‐NR024118 during the inflammatory response of RA.^12^ Consistent with our results, Yan et al^50^ have demonstrated that lncRNA XIST knockdown could suppress the inflammation in nervous tissues by reducing the levels of TNF‐α and IL‐6. Moreover, the upregulation of let‐7c has been shown to decrease the levels of TNF‐α and IL‐6.^19^ Lv et al^51^ have proposed that let‐7c‐5p can also inhibit neuroinflammation. These findings confirmed that both lncRNA XIST knockdown and let‐7c‐5p overexpression could repress inflammatory responses in RA.

In addition, the results of this study indicated that the expressions of osteogenesis‐related genes (ALP, OCN, TGF‐β1, and IGF‐1), ALP activity, and positive rate of type I collagen protein were all increased in cells transfected with sh‐lncRNA XIST or let‐7c‐5p mimic, suggesting that the silencing of lncRNA XIST and the upregulation of let‐7c‐5p both promoted osteoblast proliferation and differentiation in RA. ALP and OCN are critical markers of osteoblast differentiation, and increased levels of ALP and OCN are markers for promoted osteoblast differentiation.^52^ As one of genetic factors, TGF‐β exerts regulatory effects on osteoblasts. In fact, a high level of TGF‐β expression has been correlated to a faster function recovery in RA.^53^ Furthermore, IGF1 is regarded as a key mediator in the developmental processes, including cell proliferation and differentiation, and RA patients were associated with a low level of IGF1 expression.^54^ Type I collagen has been demonstrated as an inducer of cartilage defects.^55^ A previous study has revealed that lncRNA AK141205 exerts great effects on osteoblast differentiation by regulating ALP activity and by regulating the expression of osteogenesis‐related genes.^56^ It has been proved that the inhibition of lncRNA ANCR promoted osteoblast differentiation.^57^ Similarly, miR‐142‐3p also enhances osteoblast differentiation via the Wnt signaling pathway.^58^ Zhou et al^59^ have demonstrated that downregulated miR‐17‐92 in osteoblasts could lower the level of type I collagen, reduce the proliferation rate, and reduce ALP activity, indicating that miR‐17‐92 overexpression could increase the level of type I collagen, proliferation rate, and ALP activity.

## 5 CONCLUSIONS

In conclusion, downregulation of lncRNA XIST promoted the proliferation and differentiation of osteoblasts in RA via the inhibition of STAT3 by increasing the expression of let‐7c‐5p. Therefore, silencing of lncRNA XIST combined with increased let‐7c‐5p expression may aid the treatment of RA. However, due to the limited simple size and experimental conditions of this study, further studies are required to clarify the underlying mechanisms by which lncRNA XIST knockdown and the overexpression of let‐7c‐5p prevent the progression of RA.

## AUTHOR CONTRIBUTIONS

Zong‐Qiang Wang, Dian‐Hui Xiu, Gui‐Feng Liu, and Jin‐Lan Jiang designed the study. Gui‐Feng Liu and Jin‐Lan Jiang collated the data, carried out data analyses, and produced the initial draft of the manuscript. Zong‐Qiang Wang and Dian‐Hui Xiu contributed to drafting the manuscript. All authors have read and approved the final submitted manuscript.
